This article has been retracted.

# The impact of PEG-induced drought stress on seed germination and seedling growth of different bread wheat (*Triticum aestivum* L.) genotypes

**DOI:** 10.1371/journal.pone.0262937

**Published:** 2022-02-11

**Authors:** Shahzadi Mahpara, Aleena Zainab, Rehmat Ullah, Salma Kausar, Muhammad Bilal, Muhammad Imran Latif, Muhammad Arif, Imran Akhtar, Abdulrahman Al-Hashimi, Mohamed S. Elshikh, Marek Zivcak, Ali Tan Kee Zuan

**Affiliations:** 1 Department of Plant Breeding and Genetics, Faculty of Agricultural Sciences, Ghazi University, Dera Ghazi Khan, Pakistan; 2 Soil and Water Testing Laboratory for Research, Dera Ghazi Khan, Punjab, Pakistan; 3 Senior Scientist (Agri Chemistry), Soil and Water Testing Laboratory, Lodhran, Pakistan; 4 Scientific Officer, Soil and Water Testing Laboratory, Narowal, Pakistan; 5 Scientific Officer (Lab), Soil and Water Testing Laboratory, Layyah, Pakistan; 6 Senior Scientist (Ento), Regional Agriculture Research Institute, Bahawalpur, Pakistan; 7 Department of Botany and Microbiology, College of Science, King Saud University, Riyadh, Saudi Arabia; 8 Department of Plant Physiology, Slovak University of Agriculture, Nitra, Slovakia; 9 Department of Land Management, Faculty of Agriculture, Universiti Putra Malaysia, Selangor, Malaysia; Harran Üniversitesi: Harran Universitesi, TURKEY

## Abstract

Wheat is an important crop, used as staple food in numerous countries around the world. However, wheat productivity is low in the developing world due to several biotic and abiotic stresses, particularly drought stress. Non-availability of drought-tolerant wheat genotypes at different growth stages is the major constraint in improving wheat productivity in the developing world. Therefore, screening/developing drought-tolerant genotypes at different growth stages could improve the productivity of wheat. This study assessed seed germination and seedling growth of eight wheat genotypes under polyethylene glycol (PEG)-induced stress. Two PEG-induced osmotic potentials (i.e., -0.6 and -1.2 MPa) were included in the study along with control (0 MPa). Wheat genotypes included in the study were ‘KLR-16’, ‘B6’, ‘J10’, ‘716’, ‘A12’, ‘Seher’, ‘KTDH-16’, and ‘J4’. Data relating to seed germination percentage, root and shoot length, fresh and dry weight of roots and shoot, root/shoot length ratio and chlorophyll content were recorded. The studied parameters were significantly altered by individual and interactive effects of genotypes and PEG-induced osmotic potentials. Seed germination and growth parameters were reduced by osmotic potentials; however, huge differences were noted among genotypes. A reduction of 32.83 to 53.50% was recorded in seed germination, 24.611 to 47.75% in root length, 37.83 to 53.72% in shoot length, and 53.35 to 65.16% in root fresh weight. The genotypes, ‘J4’, ‘KLR-16’ and ‘KTDH-16’, particularly ‘J4’ better tolerated increasing osmotic potentials compared to the rest of the genotypes included in the study. Principal component analysis segregated these genotypes from the rest of the genotypes included in the study indicated that these can be used in the future studies to improve the drought tolerance of wheat crop. The genotype ‘J4’ can be used as a breeding material to develop drought resistant wheat genotypes.

## Introduction

Wheat (*Triticum aestivum* L.) belongs to Triticeae tribe and Poaceae family. It globally important cereal supposed to be originated in the Middle East region of Asia [1, 2]. Tetraploid and hexaploidy form of wheat has been domesticated since 10,000 years ago [3]. Hexaploid form is modern day bread wheat and fulfills dietary needs of the global population. The Northern India, Northern USA, and neighboring areas in Canada, Northern and Central Europe, Southern Australia, and South Africa are the major bread wheat producing areas in the world. Global population is expected to reach10 billion by 2050, which would require double of the current global food production. Expected climate changes would make the crop production difficult because of sudden changes in temperature and rainfall [4]. Wheat contributes 2% towards gross domestic product and 9.9% towards value added in agriculture. The area under wheat production in the country fluctuates within 2–5% increase or decrease due to various factors [5].

Seedling stage of crop plants is highly vulnerable to the water deficit. Seed germination is a prerequisite and important transition stage for crop plants from seeds to seedlings. The semi-arid regions of the world experience low moisture availability during seed germination of wheat crop [6]. Low moisture availability during seed germination and subsequent growth stages of wheat crop declines both production maturity time [7, 8]. The impacts of water stress on seed germination and vegetative growth of different crops such as wheat [8], maize and barley [8–10] in earlier studies. The impact of drought stress on seed germination and seedling stage of four bread wheat varieties have been evaluated and reduction in these traits was noted with significant differences among tested varieties [6, 11].

The successful establishment of crop plants relies on microclimatic conditions of seedbed and seed quality [12, 13]. Hence, seed germination of crop plants is tested under simulated environments to infer their tolerance to adverse environmental conditions. Observing seed germination under polyethylene glycol (PEG) induced drought stress is the most common screening method used to test the drought tolerance of different crop varieties during seed germination and early stand establishment [14]. Inferring changes in root length or root depth of the seedlings subjected to drought stress could provide valuable insights regarding these traits [15, 16]. Higher tolerance to adverse environmental conditions during seedling stage results in better crop production [15]. Screening a large pool of available genotypes under adverse environmental conditions is a fundamental method to select the tolerant genotypes for improved crop production. The use of osmotic substances of high molecular weight such as PEG is a common method to test the drought tolerance of crop plants during seed germination and seedling establishment [17, 18].

Seed germination and seedling emergence/establishment are important criteria for testing the tolerance of wheat genotypes to various abiotic stresses, particularly, drought stress [8, 19]. Seed germination percentage and seedling establishment are significantly reduced when soil osmotic potential reaches to -1.5 MPa [20]. Short-statured wheat cultivars have slower initial growth and their coleoptile length and leaf index undergoes decline during early growth periods [21]. Reduced coleoptile length indicates low seed germination and subsequent low plant height, whereas increased coleoptile length would result in larger initial leaf sizes and accelerate seed germination [22]. Positive correlation has been reported among seed germination and radical, plumule, coleoptile length, and dry weight of radical and plumule [23, 24].

Plant breeding concentrated on the above-ground traits for a long time, while root traits have been ignored due to several difficulties [25]. Root traits have gained significant attention during the last decade [26, 27]. Screening genotypes for early drought tolerance and inferring their root attributes at seedling stage has witnessed significant progress [28, 29]. The genotypes with higher root volume combined with longer seminal and adventitious root length has been suggested as useful candidates for increasing grain yield [30]. Plant growth, root to shoot ratio and root length could also be useful characteristics for improving the yield under arid and semi-arid climatic conditions [31, 32].

The PEG has been frequently used to for genotypes’ screening for drought tolerance at earlier growth stage. The PEG reduces seed germination and growth by reducing water potential, and the effect is observed more on the shoots compared to primary roots [13, 33]. Several studies indicated that in vitro screening using PEG is one of the reliable approaches to select drought-tolerant genotypes based on germination indices [16, 32]. The PEG is involved in the transfer of ions and nonionic compounds such as mannitol, raffinose and inulin [34, 35]. The earlier study [35] proposed that PEG is a high molecular weight non-ionic substance that is water soluble and anti-penetrable. The decrease in osmotic and water potential due to PEG has a positive correlation with the accumulation of proline which leads to decrease in osmotic stress and helps to maintain plant growth [36].

Although plenty of lines/genotypes of wheat crop are being developed on regional scales, their testing for drought tolerance at seedling stage is rarely done. Therefore, current study tested drought tolerance of eight recently developed wheat genotypes/lines in Pakistan through PEG-induced osmotic stress. It was hypothesized that the tested genotypes will differ in their drought tolerance and growth traits. It was further hypothesized that increasing negative osmotic potential would reduce seed germination and seedling traits. The results will help to select the most tolerant genotypes for breeding purposes to develop drought tolerant genotypes in the future.

## Materials and methods

### Experimental site

The current study was conducted at Plant Breeding and Genetics Laboratory, Dera Ghazi Khan, Pakistan. Eight different wheat genotypes (Table 1) with unknown drought tolerance were included in the study. There was no permit needed required to conduct the study as it did not involve any endangered species. Three different osmotic potentials, i.e., 0, -0.6 MPa and -1.2 MPa were included in the study by using PEG-6000 [37]. The desired quantity of PEG-6000 was mixed in the distilled water to make the solutions of -0.6 MPa and -1.2 MPa, whereas distilled water was used in the control treatment [37].

**Table 1:** The codes, names and drought tolerance levels of different wheat genotypes included in the study.

Genotype Code	Genotype Name	Drought tolerance
G_1_	‘KLR-16’	Unknown
G_2_	‘B6’	Unknown
G3	‘J10’	Unknown
G4	‘716’	Unknown
G5	‘A12 (Ujala)’	Unknown
G6	‘Seher’	Mild
G7	‘KTDH-16’	Unknown
G8	‘J4 (9268)’	Unknown

### Seed germination experiment

Three replicates of 25 sterilized (with 5% sodium hypochlorite) seeds were germinated between the two layers of Whatman No.1 filter paper in Petri dishes (150 × 15 mm). The 10 ml treatment solution or distilled water was poured on the filter paper and afterwards the solution or distilled water was given according to the needs. The Petri dishes were sealed with Parafilm to prevent evaporation. Seeds were incubated at 20 ± 2°C and 12 hours light dark period for 10 days. Seed germination percentage was observed every 24 hours for 10 days and then seed germination percentage was computed. The seed was considered as ‘germinated’ once the radicle elongated to 1–2 mm.

### Seedling growth experiment

Seedling growth experiment was carried out in plastic pots (97 × 165 × 90 mm) filled with a mixture of the sand and peat (1:1). The pots were placed into growth cabinet with 3 replications and 10 seeds were planted in each replication. Seeds were sown 3 cm in depth and pots irrigated with PEG-6000 solutions as to generate osmatic potentials of 0, -0.6 and -1.2 MPa. Pots were incubated under 25°C and 70–80% relative humidity for 20 days. A seed/seedling was considered as emerged when the emerging radicle reached to soil surface. Different growth traits such as root length, shoot length, fresh root weight, fresh shoot weight, dry root weight, dry shoot weight, and root, shoot ratio were measured from three weeks old seedling. The experiment was laid out according to randomized complete block design with split plot arrangements. Genotypes were considered as main factor, whereas osmotic potentials were regarded as sub-factor. The seedlings were taken off from the pots, rinsed with water to remove the debris, measured for root, and shoot lengths, divided into roots and shoots and dried in an oven (roots and shoots separately) to infer the dry weight. The chlorophyll index was measured with SPAD meter and expressed as SPAD values.

### Statistical analysis

The collected data were tested for normality, which indicated that data were normally distributed. Two-way analysis of variance (ANOVA) was then used to infer the significance in the data. Least significant difference test at 5% probability was used to compare the means where ANOVA indicated significant difference. Principal component analysis with Kaiser normalization was used to better visualize the data. The principal components with >1 eigenvalue were interpreted. Similarly, the variable having >0.60 factor loading was considered to significantly affect the relevant principal component. All computations were made on XLSTAT add-in of Microsoft Excel program. The minimal dataset of the study has been uploaded as S3 Table.

## Results

Individual and interactive effects of genotypes and PEG-induced drought stress significantly altered seed germination percentage, root and shoot length, fresh and dry weights of roots and shoot, root:shoot ratio and chlorophyll index (S1 Table). Overall, the highest seed germination percentage (78.11%) was recorded for genotype ‘J4’, whereas genotype ‘716’ resulted in the lowest (64.33%) seed germination (Table 2). Similarly, the highest (16.02 cm) and the lowest (11.72 cm) root length was noted for the genotypes ‘J4’ and ‘716’, respectively. The highest shoot length (11.98 cm), root fresh weight (0.47 g), root dry weight (0.23 g), shoot fresh weight (0.42 g), shoot dry weight (0.24 g) and chlorophyll index (49.86 SPAD value) was noted for the genotype ‘J4’. However, the lowest shoot length (8.34 cm) was recorded for the genotype ‘A12’, while the genotype ‘A12’ observed the lowest root fresh weight (0.35 g), shoot fresh weight (0.27 g), and shoot dry weight (0.10 g). Nonetheless, the lowest root dry weight (0.16 g) was recorded for the genotype ‘716’, whereas the genotype ‘Seher’ resulted in the lowest chlorophyll index (41.02 SPAD value) (Table 2).

**Table 2:** The impact of different genotypes on their seed germination and growth traits grown under different osmotic potentials.

Genotypes	GP	RL	SL	RFW	RDW	SFW	SDW	R/S	Chl
	(%)	(cm)	(cm)	(g)	(g)	(g)	(g)		(SPAD value)
**J4**	78.11 a	16.02 a	11.98 a	0.47 a	0.23 a	0.42 a	0.24 a	1.35 d	49.86 a
**KTDH-16**	73.22 b	14.58 b	10.58 b	0.43 b	0.22 a	0.36 bc	0.20 b	1.40 c	46.83 b
**KLR-16**	71.11 c	14.03 c	10.71 b	0.43 b	0.23 a	0.37 b	0.18 c	1.31 e	43.57 de
**B6**	70.55 c	13.37 d	9.62 d	0.43 b	0.23 a	0.35 cd	0.18 c	1.45 b	44.90 c
**J10**	71.22 c	12.43 e	10.05 c	0.40 c	0.20 b	0.34 d	0.16 d	1.26 f	44.13 cd
**Seher**	67.00 d	12.32 e	9.27 e	0.39 cd	0.18 c	0.34 d	0.17 d	1.34 d	41.02 f
**A12**	66.66 d	12.27 e	8.34 f	0.38 d	0.16 d	0.28 e	0.11 e	1.52 a	46.55 b
**716**	64.33 e	11.72 f	9.04 e	0.35 e	0.17 c	0.27 e	0.10 e	1.30 e	42.86 e
**LSD 5%**	1.01	0.22	0.25	0.09	0.013	0.015	0.01	0.24	0.85

Here, GP = seed germination percentage, RL = root length, SL = shoot length, RFW = root fresh weight, RDW = root dry weight, SFW = shoot fresh weight, SDW = shoot dry weight, R/S = root:shoot ratio, Chl = chlorophyll index. The means sharing same letters within a same column are statistically non-significant (p > 0.05).

The highest values of seed germination percentage, root and shoot length, fresh and dry weights of roots and shoot, and chlorophyll index were recorded for control treatment, whereas the lowest values of these traits were noted for -1.2 MPa osmotic potential (Table 3). Contrastingly, the highest root:shoot ratio was noted for -0.6 MPa osmotic potential, whereas the lowest value was noted under control treatment of the study (Table 3).

**Table 3:** The impact of different osmotic potentials on seed germination and growth traits of different wheat genotypes included in the study.

Osmotic potential	GP	RL	SL	RFW	RDW	SFW	SDW	R/S	Chl
	(%)	(cm)	(cm)	(g)	(g)	(g)	(g)		(SPAD value)
**0 MPa**	100.00 a	18.34 a	14.55 a	0.69 a	0.31 a	0.60 a	0.30 a	1.27 c	49.44 a
**-0.6 MPa**	70.08 b	13.97 b	9.79 b	0.37 b	0.21 b	0.30 b	0.15 b	1.43 a	45.53 b
**-1.2 MPa**	40.75 c	7.72 c	5.50 c	0.17 c	0.08 c	0.12 c	0.05 c	1.41 b	39.92 c
**LSD 5%**	0.62	0.13	0.15	0.015	0.008	0.009	0.006	0.013	0.52

Here, GP = seed germination percentage, RL = root length, SL = shoot length, RFW = root fresh weight, RDW = root dry weight, SFW = shoot fresh weight, SDW = shoot dry weight, R/S = root:shoot ratio, Chl = chlorophyll index. The means sharing same letters within a same column are statistically non-significant (p > 0.05).

Regarding genotypes by drought stress interaction, all genotypes resulted in 100% seed germination under control treatment; however, seed germination recorded a significant decrease. The genotype ‘J4’ with control treatment recorded the highest values for seed germination percentage, root and shoot length, fresh and dry weights of roots and shoot, and chlorophyll index, whereas the lowest values for these traits were noted for the genotypes ‘716’ an ‘A12’ germinated under -1.2 MPa osmotic potential (Table 4). The genotypes ‘J4’ and ‘KTDH-16’ better tolerated increasing level of drought stress compared to the rest of the treatments included in the study, whereas genotypes ‘716’ and ‘A12’ proved as the most sensitive genotypes.

**Table 4:** The impact of wheat genotypes by different osmotic potentials’ interaction on seed germination and growth traits of wheat genotypes included in the study.

Interactions	GP	RL	SL	RFW	RDW	SFW	SDW	R/S	Chl
	(%)	(cm)	(cm)	(g)	(g)	(g)	(g)		(SPAD value)
**G**_**1**_ **× O**_**1**_	100.00 a	17.20 d	13.73 d	0.54 e	0.28 ef	0.48 f	0.17 g	1.25 gh	47.50 de
**G**_**2**_ **× O**_**1**_	100.00 a	17.50 d	13.00 e	0.65 d	0.26 fg	0.53 e	0.23 e	1.34 ef	52.66 ab
**G**_**3**_ **× O**_**1**_	100.00 a	18.46 c	14.03 cd	0.72 b	0.32 bc	0.64 c	0.33 c	1.33 ef	49.40 c
**G**_**4**_ **× O**_**1**_	100.00 a	17.13 d	14.36 c	0.68 c	0.30 cd	0.61 d	0.30 d	1.19 i	51.66 b
**G**_**5**_ **× O**_**1**_	100.00 a	19.16 b	16.03 a	0.76 a	0.37 a	0.69 a	0.38 a	1.22 h	53.53 a
**G**_**6**_ **× O**_**1**_	100.00 a	19.46 ab	15.66 ab	0.72 b	0.33 b	0.62 cd	0.31 d	1.24 h	46.73 ef
**G**_**7**_ **× O**_**1**_	100.00 a	19.66 a	15.43 b	0.75 a	0.36 a	0.66 b	0.36 b	1.28 g	48.66 cd
**G**_**8**_ **× O**_**1**_	100.00 a	18.13 c	14.20 c	0.70 bc	0.28 de	0.62 cd	0.31 cd	1.28 g	45.40 fg
**G**_**1**_ **× O**_**2**_	59.66 g	11.50 i	8.73 i	0.34 jk	0.17 k	0.24 j	0.09 i	1.32 f	43.00 hi
**G**_**2**_ **× O**_**2**_	62.00 f	12.26 h	7.93 j	0.33 k	0.19 jk	0.24 j	0.07 j	1.58 b	46.40 ef
**G**_**3**_ **× O**_**2**_	70.66 d	13.46 g	9.36 h	0.36 ij	0.22 hi	0.29 i	0.16 g	1.45 d	45.66 f
**G**_**4**_ **× O**_**2**_	71.00 d	13.10 g	10.33 g	0.35 ijk	0.20 ij	0.29 i	0.13 h	1.25 gh	43.03 hi
**G**_**5**_ **× O**_**2**_	82.00 b	18.36 c	12.33 f	0.42 f	0.24 g	0.38 g	0.23 e	1.48 c	52.40 ab
**G**_**6**_ **× O**_**2**_	67.66 e	14.43 f	10.30 g	0.39 gh	0.24 gh	0.33 h	0.16 g	1.36 e	44.16 gh
**G**_**7**_ **× O**_**2**_	75.66 c	16.03 e	10.20 g	0.40 fg	0.25 g	0.34 h	0.20 f	1.57 b	50.00 c
**G**_**8**_ **× O**_**2**_	72.00 d	12.63 h	9.16 hi	0.37 hi	0.21 ij	0.33 h	0.17 g	1.41 d	39.63 k
**G**_**1**_ **× O**_**3**_	33.33 m	6.46 m	4.66 m	0.16 o	0.08 m	0.11 n	0.04 l	1.32 f	38.10 l
**G**_**2**_ **× O**_**3**_	38.00 l	7.06 l	4.10 n	0.17 o	0.03 n	0.06 p	0.02 lm	1.66 a	40.60 jk
**G**_**3**_ **× O**_**3**_	41.00 k	8.20 k	5.46 l	0.22 lm	0.15 l	0.13 m	0.06 jk	1.58 b	39.63 k
**G**_**4**_ **× O**_**3**_	42.66 jk	7.06 l	5.45 l	0.18 no	0.10 m	0.14 lm	0.07 j	1.34 ef	37.70 l
**G**_**5**_ **× O**_**3**_	52.33 h	10.53 j	7.60 j	0.24 l	0.08 m	0.19 k	0.11 h	1.35 ef	43.66 h
**G**_**6**_ **× O**_**3**_	45.66 i	8.20 k	6.16 k	0.19 mn	0.13 l	0.16 l	0.09 i	1.34 ef	39.83 k
**G**_**7**_ **× O**_**3**_	44.00 ij	8.06 k	6.13 k	0.13 p	0.05 n	0.10 no	0.04 kl	1.34 ef	41.83 ij
**G**_**8**_ **× O**_**3**_	29.00 n	6.20 m	4.46 mn	0.12 p	0.04 n	0.08 op	0.01 m	1.32 f	38.03 l
**LSD 5%**	1.76	0.39	0.44	0.027	0.022	0.023	0.017	0.037	1.48

Here, G_1_ = 716, G_2_ = A12, G_3_ = B6, G_4_ = J10, G_5_ = J4, G_6_ = KLR-16, G_7_ = KTDH16, G_8_ = Seher, O_1_ = control (0 MPa), O_2_ = -0.6 MPa, O_3_ = -1.2 MPa. Here, GP = seed germination percentage, RL = root length, SL = shoot length, RFW = root fresh weight, RDW = root dry weight, SFW = shoot fresh weight, SDW = shoot dry weight, R/S = root:shoot ratio, Chl = chlorophyll index. The means sharing same letters within a same column are statistically non-significant (p > 0.05).

The decrease in seed germination percentage, root and shoot length, fresh and dry weights of roots and shoot, and chlorophyll index, and increase in root:shoot ratio was significantly altered by individual and interactive effects of genotypes and PEG-induced drought stress levels (S2 Table). Overall, the highest decrease in seed germination percentage (53.50%) and root length (45.75%) was recorded for genotype ‘716’, whereas genotype ‘J4’ recorded the lowest decline in these traits compared to the rest of the genotypes included in the study (Table 5). The genotype ‘A12’ observed the highest decrease in shoot length, root dry weight, shoot fresh weight and shoot dry weight. The lowest decrease in these traits was recorded for the genotype ‘J4’. Similarly, genotypes ‘716’ and ‘Seher’ observed the highest increase in root:shoot ratio, whereas the lowest increase was noted for genotype ‘A12’ (Table 5).

**Table 5:** The impact of different genotypes on percentage decrease in their seed germination and growth traits under different osmotic potentials.

Genotypes	GP	RL	SL	RFW	RDW	SFW	SDW	R/S *	Chl
	(%)	(cm)	(cm)	(g)	(g)	(g)	(g)		(SPAD value)
**716**	53.50 a	47.75 a	51.21 b	53.35 c	54.19 b	62.82 de	61.67 c	6.05 a	14.59 bc
**A12**	50.00 b	44.75 b	53.72 a	61.19 b	56.37 ab	71.37 a	79.23 a	20.80 c	17.38 b
**B6**	44.16 c	41.33 c	47.15 c	59.64 b	42.21 d	66.40 bc	66.66 b	14.03 b	13.65 c
**J10**	43.16 c	41.14 c	45.05 c	61.03 b	50.05 c	64.22 cd	66.60 b	9.40 a	21.87 a
**J4**	32.83 e	24.61 e	37.83 d	56.09 c	55.37 ab	58.44 f	54.78 d	16.08 b	10.27 d
**KLR-16**	43.33 c	41.86 c	47.45 c	59.63 b	43.46 d	60.50 ef	58.59 cd	9.19 a	10.11 d
**KTDH-16**	40.16 d	38.73 d	47.07 c	64.35 a	58.30 a	66.80 b	66.199b	13.43 b	5.62 e
**Seher**	49.50 b	48.06 a	51.99 ab	65.16 a	54.60 b	67.04 b	69.51 b	6.667a	14.46 c
**LSD 5%**	1.54	1.76	2.45	2.87	3.63	2.35	4.05	3.48	2.91

Here, GP = seed germination percentage, RL = root length, SL = shoot length, RFW = root fresh weight, RDW = root dry weight, SFW = shoot fresh weight, SDW = shoot dry weight, R/S = root:shoot ratio, Chl = chlorophyll index. The means sharing same letters within a same column are statistically non-significant (p > 0.05).

* indicated that relevant trait was increased instead of decrease

The highest decrease in seed germination percentage, root and shoot length, fresh and dry weights of roots and shoot, and chlorophyll index was recorded for -1.2 MPa osmotic potential compared to the control treatment of the study, whereas the lowest decrease was recorded for -0.6 MPa osmotic potential (Table 6). The root:shoot ratio was not altered by the osmotic potentials included in the study (Table 6).

**Table 6:** The impact of different osmotic potentials on percentage decrease in their seed germination and growth traits under different osmotic potentials.

Osmotic potential	GP	RL	SL	RFW	RDW	SFW	SDW	R/S*	Chl
	(%)	(cm)	(cm)	(g)	(g)	(g)	(g)		(SPAD value)
**-0.6 MPa**	29.91 b	24.05 b	32.92 b	45.96 b	30.59 b	49.47 b	50.00 b	12.80	7.88 b
**-1.2 MPa**	59.25 a	58.00 a	62.45 a	74.15 a	73.04 a	79.93 a	80.81 a	11.11	19.10 a
**LSD 5%**	0.77	0.59	1.22	1.43	1.81	1.17	2.02	NS	1.45

Here, GP = seed germination percentage, RL = root length, SL = shoot length, RFW = root fresh weight, RDW = root dry weight, SFW = shoot fresh weight, SDW = shoot dry weight, R/S = root:shoot ratio, Chl = chlorophyll index. The means sharing same letters within a same column are statistically non-significant (p > 0.05).

* indicated that relevant trait was increased instead of decrease

Regarding genotypes by drought stress interaction, the genotype ‘Seher’ with -1.2 MPa treatment recorded the highest decrease in seed germination percentage, root and shoot length, fresh and dry weights of roots and shoot, and chlorophyll index, whereas the lowest decrease in these traits were noted for the genotypes ‘J4’ under -0.6 MPa osmotic potential (Table 7). The genotypes ‘J4’ and ‘KTDH-16’ better tolerated increasing level of drought stress compared to the rest of the treatments included in the study, whereas genotypes ‘Seher’, ‘716’ and ‘A12’ proved as the most sensitive genotypes.

**Table 7:** The impact of wheat genotypes by different osmotic potentials’ interaction on decrease in seed germination and growth traits of wheat genotypes included in the study.

Interactions	GP	RL	SL	RFW	RDW	SFW	SDW	R/S	Chl
	(%)	(cm)	(cm)	(g)	(g)	(g)	(g)		(SPAD value)
**G**_**1**_ **× O**_**2**_	40.33 h	33.12 f	36.38 de	37.37 h	38.08 f	48.61 fg	47.04 gh	6.01 a-d	9.43 gh
**G**_**2**_ **× O**_**2**_	38.00 i	29.88 g	38.97 d	48.39 f	26.64 hi	54.57 e	70.03 e	17.81 fg	11.87 fg
**G**_**3**_ **× O**_**2**_	29.33 k	27.07 h	33.26 e	49.70 f	30.85 gh	54.15 e	51.45 fg	9.01 b-e	7.55 h
**G**_**4**_ **× O**_**2**_	29.00 k	23.54 i	28.05 f	48.53 f	33.73 fg	51.38 ef	56.59 f	5.64 abc	16.70 cde
**G**_**5**_ **× O**_**2**_	18.00 m	4.17 k	23.07 g	44.04 g	33.30 fg	44.25 h	40.00 i	21.46 gh	2.12 i
**G**_**6**_ **× O**_**2**_	32.33 j	25.85 h	34.26 e	46.32 fg	26.30 hi	46.80 gh	46.21 gh	10.13 cde	5.47 hi
**G**_**7**_ **× O**_**2**_	24.33 l	18.47 j	33.90 e	45.94 fg	30.31 ghi	48.67 fg	44.41 hi	22.14 gh	-2.77 j
**G**_**8**_ **× O**_**2**_	28.00 k	30.33 g	35.44 e	47.39 fg	25.53 i	47.36 gh	44.24 hi	10.19 cde	12.71 efg
**G**_**1**_ **× O**_**3**_	66.66 b	62.38 b	66.04 a	69.33 de	70.29 c	77.04 bc	76.30 cd	6.10 a-d	19.76 bc
**G**_**2**_ **× O**_**3**_	62.00 c	59.62 c	68.46 a	73.99 b	86.11 a	88.18 a	88.44 b	23.78 h	22.90 b
**G**_**3**_ **× O**_**3**_	59.00 d	55.58 d	61.04 b	69.58 cde	53.57 e	78.65 b	81.86 c	19.05 gh	19.75 bc
**G**_**4**_ **× O**_**3**_	57.33 de	58.75 c	62.05 b	73.53 bc	66.36 c	77.06 bc	76.61 cd	13.16 ef	27.03 a
**G**_**5**_ **× O**_**3**_	47.66 g	45.04 e	52.59 c	68.14 e	77.43 b	72.62 d	69.56 e	10.70 de	18.42 cd
**G**_**6**_ **× O**_**3**_	54.33 f	57.86 c	60.63 b	72.94 bcd	60.61 d	74.20 cd	70.98 de	8.24 b-e	14.70 def
**G**_**7**_ **× O**_**3**_	56.00 ef	58.98 c	60.25 b	82.76 a	86.29 a	84.93 a	87.95 b	4.72 ab	14.02 ef
**G**_**8**_ **× O**_**3**_	71.00 a	65.80 a	68.54 a	82.92 a	83.67 a	86.72 a	94.78 a	3.14 a	16.20 cde
**LSD 5%**	2.18	2.52	3.46	4.06	5.14	3.32	5.73	4.93	4.12

Here, G_1_ = 716, G_2_ = A12, G_3_ = B6, G_4_ = J10, G_5_ = J4, G_6_ = KLR-16, G_7_ = KTDH16, G_8_ = Seher, O_2_ = -0.6 MPa, O_3_ = -1.2 MPa. Here, GP = seed germination percentage, RL = root length, SL = shoot length, RFW = root fresh weight, RDW = root dry weight, SFW = shoot fresh weight, SDW = shoot dry weight, R/S = root:shoot ratio, Chl = chlorophyll index. The means sharing same letters within a same column are statistically non-significant (p > 0.05).

* indicates that the relevant trait was increased instead of decrease

Principal component analysis executed on germination and growth traits of different genotypes yielded in two principal components (PCs) with eigenvalues >1 (Table 8). The first two PCs collectively explained 91.86% variability in the dataset. The first PC was positively influenced by all measured traits except root:shoot ratio, whereas the second PC was positively affected by root:shoot ratio and chlorophyll index (Table 8).

**Table 8:** Eigenvalues, variability and factor loadings of first two principal components of principal component analysis executed on seed germination and growth traits of wheat genotypes included in the study.

Traits	PC1	PC2
**Eigenvalue**	6.76	1.50
**Variability (%)**	75.10	16.75
**Cumulative %**	75.10	91.86
**Factor loadings**		
**GP**	**0.91**	-0.03
**RL**	**0.99**	0.05
**SL**	**0.94**	-0.28
**FRW**	**0.96**	-0.05
**DRW**	**0.89**	-0.28
**FSW**	**0.99**	-0.05
**DSW**	**0.96**	0.08
**R/S**	0.11	**0.93**
**CHL**	**0.61**	**0.66**

Here, GP = seed germination percentage, RL = root length, SL = shoot length, RFW = root fresh weight, RDW = root dry weight, SFW = shoot fresh weight, SDW = shoot dry weight, R/S = root:shoot ratio, Chl = chlorophyll index. The bold values indicate that the relevant trait significantly affected the corresponding principal component

The biplot of first two PCs divided the genotypes in two major groups. The first group had three genotypes having similar seed germination percentage and growth-related traits, whereas the second group was not influenced by any studied traits. The first group contained the genotypes with higher drought tolerance while the second group included the genotypes with the lowest drought tolerance recorded in the current study (Fig 1).

**Fig 1:** Biplot of the first two principal components of principal component analysis executed on seed germination and growth traits of wheat genotypes included in the study. Here, GP = seed germination percentage, RL = root length, SL = shoot length, RFW = root fresh weight, RDW = root dry weight, SFW = shoot fresh weight, SDW = shoot dry weight, R/S = root:shoot ratio, Chl = chlorophyll index.

Principal component analysis executed on reductions in seed germination and growth traits of different genotypes in three PCs with eigenvalues >1 (Table 9). The first three PCs collectively explained 84.72% variability in the dataset. The first PC was positively influenced by seed germination percentage, root and shoot length and fresh and dry weight of root. The second PC was positively affected by root:shoot ratio and negatively affected by fresh and dry weight of root (Table 9) The third PC was only positively influenced by chlorophyll index.

**Table 9:** Eigenvalues, variability, and factor loadings of first two principal components of principal component analysis executed on percentage decrease in seed germination and growth traits of wheat genotypes included in the study.

	PC1	PC2	PC3
**Eigenvalue**	4.23	2.36	1.024
**Variability (%)**	47.09	26.25	11.37
**Cumulative %**	47.09	73.32	84.72
**Factor loadings**			
**GP**	**0.82**	0.47	0.03
**RL**	**0.84**	0.46	-0.20
**SL**	**0.89**	0.18	-0.20
**FRW**	0.52	**-0.69**	-0.23
**DRW**	0.08	**-0.67**	-0.34
**FSW**	**0.82**	-0.53	-0.03
**DSW**	**0.86**	-0.36	0.25
**R/S**	0.17	**0.70**	-0.48
**CHL**	0.54	0.19	**0.68**

Here, GP = seed germination percentage, RL = root length, SL = shoot length, RFW = root fresh weight, RDW = root dry weight, SFW = shoot fresh weight, SDW = shoot dry weight, R/S = root:shoot ratio, Chl = chlorophyll index. The bold values indicate that the relevant trait significantly affected the corresponding principal component

The biplot of first two PCs divided the genotypes in two major groups. The first group had three genotypes having similar values for decrease in seed germination percentage and growth-related traits, whereas the second group was not influenced by the decrease studied traits. The first group contained the genotypes with the lowest drought tolerance while the second group included the genotypes with the highest drought tolerance recorded in the current study (Fig 2).

**Fig 2:** Biplot of the first two principal components of principal component analysis executed on percentage decrease in seed germination and growth traits of wheat genotypes included in the study. Here, GP = seed germination percentage, RL = root length, SL = shoot length, RFW = root fresh weight, RDW = root dry weight, SFW = shoot fresh weight, SDW = shoot dry weight, R/S = root:shoot ratio, Chl = chlorophyll index.

## Discussion

Different genotypes significantly differed for their tolerance to PEG-induced drought stress as hypothesized. Similarly, the highest reduction in seed germination and growth traits was recorded under -1.2 MPa osmotic potential level compared to the control treatment of the study which supported our second hypothesis [14, 38]. Seed germination is an important transition stage from seeds to seedlings for crop plants and higher seed germination under stressful and benign environmental conditions enable plants to thrive and produce higher yields under adverse as well as benign environments [38]. Seed germination is controlled by the microclimatic conditions of the seedbed as well genetic potential of the crop plants. Genotypes by environment interactions is significant for getting higher crop yields. The semi-arid regions of the world experience low moisture availability during seed germination of wheat crop. Low moisture availability during seed germination crop declines both production maturity time [7, 8]. The impacts of water stress on seed germination and vegetative growth of different crops such as wheat [8], maize and barley [8–10] has been reported in earlier studies and a constant decline in the germination was recorded. The impact of drought stress on seed germination and seedling stage of four bread wheat varieties have been evaluated and reduction in these traits was noted with significant differences among tested varieties [11].

Seed germination is controlled by several necessary enzymes and stored food for the growing embryo. The increasing negative osmotic potential disrupts the activities of these enzymes; thus, seeds lose their germination potential [39]. The other major reason of decreased seed germination is lower imbibition of water and the moisture needs of the seeds required for seed germination are not fulfilled. The reduced seed germination under higher negative osmotic potential in the current study is linked with lower water imbibition and subsequently reduced enzyme activities necessary for seed germination. Several earlier studies have reported that increasing osmotic potential have lowered seed germination of crop plants and weed species. The tested genotypes significantly differed for their drought tolerance and the genotype ‘J4’ proved the most tolerant one compared to the rest of the genotypes included in the study. The differences among genotypes are owed to their genetic make-up as well as ability to uptake moisture necessary for the seed germination. The genotype ‘J4’ is a potential candidate for developing drought tolerant wheat varieties through conventional breeding [40].

Different growth traits of the tested genotypes were also significantly altered by the osmotic potentials used in the current study. Like seed germination, genotype ‘J4’ better tolerated moisture deficiency compared to the rest of the genotypes included in the study. The decreased growth traits under higher drought stress level can be explained with the lower moisture availability and subsequent lower transport of photosynthate from source to the sink. The differences among genotypes are owed to their inherent genetic makeup [41, 42].

Earlier studies [43, 44] have reported under water deficit reduced root length, shoot length, root weight, shoot weight, number of spike, number of grains number/spike, 1000-grain, weight and grain yield of wheat genotypes. Under drought stress root growth is limited but shoot growth is abruptly decreased [45]. The root:shoot ratio was increased in the current study indicating that all the tested genotypes tended to increase their root length under low moisture availability. However, the increased root length could not compensated the damaged caused by low water availability to growth traits [46, 47]. Chlorophyll concentration has been reported to decrease under drought stress [24, 48] and similar was recorded in the current study.

Generally, G × PEG-induced drought stress interactions reduced germinations and seedling characteristics of the studied genotypes. The PCA divided the genotypes into 2 distinct groups, i.e., group 1 and group 2 according to seed germination growth traits and decrease in seed germination and growth traits were tolerant to drought stress compared to the rest of the genotypes included in the study. Thus, the identified genotypes, particularly, ‘J4’ can be used for improving drought tolerance of bread wheat genotypes [49].

## Conclusion

Different genotypes significantly differed for their tolerance to PEG-induced drought stress as hypothesized. Similarly, the highest reduction in seed germination and growth traits was recorded under -1.2 MPa osmotic potential level compared to the control treatment of the study which supported our second hypothesis. The genotype ‘J4’ better tolerated drought stress compared to the rest of the genotypes included in the study. Therefore, ‘J4’ can be used as breeding material to improve drought tolerance of wheat crop.

## Supporting information

S1 Table Analysis of variance for seed germination percentage and growth traits of different wheat genotypes grown under various PEG-induced drought stress levels. (DOCX)

S2 Table Analysis of variance for percentage decrease in seed germination percentage and growth traits of different wheat genotypes grown under various PEG-induced drought stress levels. (DOCX)

S3 Table Minimal dataset used in the study to build graphs and perform statistical analysis. (XLSX)
